The article "A Clinical Diagnostic Value Analysis of Serum CA125, CA199, and HE4 in Women with Early Ovarian Cancer: Systematic Review and Meta-Analysis" was retracted in 2023. Reasons: unreliable results or conclusions; concerns about the data; concerns about the peer review; concerns about the citations.

# A Clinical Diagnostic Value Analysis of Serum CA125, CA199, and HE4 in Women with Early Ovarian Cancer: Systematic Review and Meta-Analysis

**DOI:** 10.1155/2022/9339325

**Published:** 2022-05-25

**Authors:** Xiaolin Qing, Liting Liu, Xiguang Mao

**Affiliations:** ^1^Obstetrics and Gynecology, Department of Clinical College of Medicine, Southwest Medical University, China; ^2^Gynecology Department of Traditional Chinese Medicine, Affiliated Hospital of Southwest Medical University, China

## Abstract

**Objective:**

To evaluate the value of combined detection of serum CA125, CA199, and HE4 in the diagnosis of ovarian cancer.

**Methods:**

Relevant articles retrieved from PubMed, Elsevier Science, Springer, China National Knowledge Infrastructure (CNKI), Wanfang, and VIP databases were screened strictly according to inclusion and exclusion criteria. Included literature published from January 2005 to December 2021. (2) Serum HE4, CA125, CA199, and their combination for ovarian cancer diagnostic tests were studied, and healthy subjects or patients with the benign disease were taken as a control group. (3) Pathological tissue diagnosis as the gold standard. (4) Complete original data can be obtained. (5) The sample size was ≥20. (6) Language is limited to Chinese and English. Data features and QUADAS table were extracted from the included literature, and QUADAS evaluation tool detail table was used for the included study. Conduct quality evaluation. Statistical analysis was carried out using meta-disc software version 1.4. Appropriate effect model was selected to merge the effect size, and the forest maps of merge sensitivity, merge specificity, and merge likelihood ratio were obtained.

**Results:**

The results of meta-analysis showed that there was a statistical difference in diagnostic specificity analysis of CA125 (OR = 1.91, 95% CI (1.58, 2.32), *P* < 0.00001, *I*^2^ = 67%, *Z* = 6.58); diagnostic sensitivity analysis of CA125 (OR = 2.50, 95% CI (1.73, 3.62), *P* < 0.00001, *I*^2^ = 0%, *Z* = 4.90); diagnostic specificity analysis of CA199 (OR = 1.98, 95% CI (1.60, 2.44), *P* < 0.00001, *I*^2^ = 89%, *Z* = 6.35); diagnostic sensitivity analysis of CA199 (OR = 1.92, 95% CI (1.46, 2.52), *P* < 0.00001, *I*^2^ = 73%, *Z* = 4.70); diagnostic specificity analysis of HE4 (OR = 2.08, 95% CI (1.65, 2.63), *P* < 0.00001, *I*^2^ = 73%, *Z* = 6.19); diagnostic sensitivity analysis of HE4 (OR = 2.37, 95% CI (1.87, 3.00), *P* < 0.00001, *I*^2^ = 83%, *Z* = 7.19).

**Conclusion:**

In the clinical assisted diagnosis of ovarian cancer, combined detection of CA125, CA199, and HE4 has the stronger discriminant ability and higher accuracy than single detection of CA125, which can improve the diagnostic efficiency.

The article "A Clinical Diagnostic Value Analysis of Serum CA125, CA199, and HE4 in Women with Early Ovarian Cancer: Systematic Review and Meta-Analysis" was retracted in 2023. Reasons: unreliable results or conclusions; concerns about the data; concerns about the peer review; concerns about the citations.

## 1. Introduction

In the female reproductive system, ovarian cancer has become one of the three common malignant tumors, and about 85%-90% of ovarian malignant tumors are epithelial ovarian cancer [1]. In recent years, the incidence of ovarian cancer has shown a gradually increasing trend [2]. Due to the lack of early symptoms of ovarian cancer and the lack of early screening and diagnosis, the survival rate of patients has been less than 30% [3]. However, if detected at early stage and given standard surgery and adjuvant therapy, the 5-year survival rate of ovarian cancer can be as high as 90% [4]. 80% of patients with ovarian epithelial carcinoma showed the elevated expression level of carbohydrate antigen 125 (CA125) in serum, and more than 90% of patients showed serum CA125 level correlated with disease severity. HE4 is a protease inhibitor associated with sperm maturation. It was first found in human distal epididymis epithelial cells. Later studies confirmed that HE4 was not expressed in the female ovarian surface epithelium [5]. Among various tumor tissues, ovarian cancer has the highest HE4 expression level. Detection of serum HE4 is of great value for the diagnosis and monitoring of ovarian cancer.

HE4 was highly expressed in many tumors, including ovarian serous carcinoma, lung adenocarcinoma, squamous cell carcinoma, endometrial carcinoma, breast adenocarcinoma, and mesothelioma [6]. HE4 is also moderately or highly expressed in gastrointestinal tumors, kidney, and transitional cell carcinoma. HE4 is lowly expressed in prostate cancer and all liver cancers. There is an immune response in pancreatic, gallbladder, and bile duct cancers. Some studies have found that the serum concentration of HE4 is not only closely related to ovarian cancer tissue type and pathological stage but also related to age and menopausal status [7].

The expression of CA125 is associated with multiple systemic tumors (ovarian cancer, digestive system malignancy, tongue cancer, breast cancer, lung cancer, et al.). A large number of studies [8, 9] have reported that serum CA125 expression level varies in different ovarian cancer tissue types and surgical pathological stages, and the critical value of diagnosis is CA125 > 35 U/mL. A study showed that the serum CA125 in patients with ovarian epithelial cancer was significantly higher than that in germ cell tumor and sex cord-stromal tumor groups. CA125 aqueous was significantly higher in serous cystadenocarcinoma than in mucinous cystadenocarcinoma and clear cell carcinoma.

CA199 is a kind of mucosal glycoprotein, mainly secreted by tumor cells of the digestive tract. At present, CA199 is also used as a marker of gynecological tumors in combination with other tumor markers. As a soluble glycoprotein with a complex substance structure, HE4 is a nonspecific tumor marker, which is also expressed in different degrees in cervical cancer, endometrial cancer, ovarian epithelial, and nonepithelial cancers, in addition to colorectal cancer and gastrointestinal malignancies [10]. Its content is correlated with tumor size and metastasis. Continuous detection of its content in blood and other body fluids can provide a basis for differential diagnosis and prognosis of the disease.

The article "A Clinical Diagnostic Value Analysis of Serum CA125, CA199, and HE4 in Women with Early Ovarian Cancer: Systematic Review and Meta-Analysis" was retracted in 2023. Reasons: unreliable results or conclusions; concerns about the data; concerns about the peer review; concerns about the citations.

A large number of studies have reported that combination of serum HE4, CA199, and CA125 can be used for diagnostic in ovarian cancer, but the specificity and sensitivity of these serum tumor markers are still controversial. Therefore, this study systematically reviewed the application of serum HE4, CA199, and CA125 in the diagnostic of ovarian cancer and will bring up new lights for the treatment in ovarian cancer.

## 2. Materials and Methods

### 2.1. Inclusion Criteria

(1) Included literature published from January 2005 to December 2021. (2) Serum HE4, CA125, CA199, and their combination for ovarian cancer diagnostic tests were studied; and healthy subjects or patients with the benign disease were taken as a control group. (3) Pathological tissue diagnosis as the gold standard. (4) Complete original data can be obtained. (5) The sample size was ≥20. (6) Language is limited to Chinese and English. About 3 reviewers screened each record and the reviewers worked independently.

### 2.2. Exclusion Criteria

1. The content of the study only described the diagnostic value of serum HE4, CA125, CA199, and their combined application for ovarian cancer, but there was no descriptive study of the control group; (2) ovarian cancer patients with a history of surgery or antineoplastic therapy; (3) literature with incorrect calculation and incomplete data; (4) conference, lecture, review, abstract, and review literature; (5) use the same data or duplicate publications.

### 2.3. Retrieval Strategy

PubMed, Elsevier Science, Springer, CNKI, Wanfang, VIP, and other databases were searched by computer. Literature languages are limited to Chinese and English. HE4 and CA125 and ovarian cancer; hE4; ovarian cancer; serum biomarkers; diagnosis, etc. as search terms (Figure 1).

### 2.4. Extraction of Literature

This study by two people as evaluators, in strict accordance with the inclusion criteria and exclusion criteria to an independent screening of literature, respectively, after extracting data to cross-check, ensures the quality of literature to extract and review price is the consistency of the results when disagreements are resolved through discussion, as there are still differences through consulting a guidance group of other experts to solve. Extracted data include author, age, country, test method, positive determination value, gold standard, and fruit index.

The article "A Clinical Diagnostic Value Analysis of Serum CA125, CA199, and HE4 in Women with Early Ovarian Cancer: Systematic Review and Meta-Analysis" was retracted in 2023. Reasons: unreliable results or conclusions; concerns about the data; concerns about the peer review; concerns about the citations.

### 2.5. Data Extraction

The studies included in this paper were all diagnostic test accuracy studies, and their quality was evaluated from the following aspects: (1) whether the case spectrum included various medical records and cases of easily confused diseases; (2) whether the criteria for the selection of research objects are clear; (3) whether the clinical data available when interpreting test results are consistent with the clinical data available in practice; (4) whether intermediate test results are reported; (5) whether to explain the cases that withdrew from the study.

### 2.6. Literature Bias Analysis

*x* ^2^ test was used to analyze the heterogeneity among the included studies. The test was quasiset as 0.05. If the heterogeneity between studies could not be eliminated by processing. Heterogeneity can be evaluated by *I*^2^, and small heterogeneity is <25%, medium heterogeneity is represented by 25-50%, and when there is high heterogeneity between the results, it is represented by >50%. Whether the random effect model or the fixed effect model is used to summarize accuracy indicators depends on the heterogeneity, and the fixed effect model is used for those with low heterogeneity. The source of heterogeneity in this paper can be discussed by meta-regression analysis. After selecting the effect model, all effect sizes were calculated and combined (Figures 2 and 3).

### 2.7. Statistical Analysis

The heterogeneity among the included studies was analyzed. The threshold effect is one of the main reasons for the heterogeneity of accurate research. The meta-disc soft piece can be used to evaluate the threshold effect by three methods: view test, spearman correlation coefficient calculation, and the image generated by the exact estimator of each study in the SROC curve plan. Interstudy heterogeneity can be caused by nonthreshold effects, such as differences in subjects, differences in test criteria and conditions, reference criteria, interstudy design, and implementation methods. MetaDisc1.4 software provides two methods to evaluate heterogeneity caused by nonthreshold effects: observed forest maps and statistical tests, including chi-square test and Cochran-Q.

## 3. Result

### 3.1. Literature Retrieval Results and Basic Features of Included Studies

After screening, a total of 15 studies were finally included [11–24]. All the included studies were diagnostic tests, including 2262 patients with ovarian cancer, all confirmed by national pathological standards, and the control group included 2300 patients with benign ovarian disease and healthy people, and a total of 4562 cases were included. The basic characteristics included in the study are shown in Table 1.

The article "A Clinical Diagnostic Value Analysis of Serum CA125, CA199, and HE4 in Women with Early Ovarian Cancer: Systematic Review and Meta-Analysis" was retracted in 2023. Reasons: unreliable results or conclusions; concerns about the data; concerns about the peer review; concerns about the citations.

### 3.2. Diagnostic Specificity Analysis of CA125

Among the 15 research literatures, no threshold effect was caused by high heterogeneity. The results of the forest Figures 4–9 showed that the effects of the amount of ci had little or no overlap. Within these few studies, the heterogeneity markedly improved were excluded, and random effect model was used to analyze the mining meta. The difference in diagnostic specificity analysis of CA125 between the two groups was statistically significant (OR = 1.91, 95% CI (1.58, 2.32), *P* < 0.00001, *I*^2^ = 67%, *Z* = 6.58).

### 3.3. Diagnostic Sensitivity Analysis of CA125

The difference in diagnostic sensitivity analysis of CA125 between the two groups was statistically significant (OR = 2.50, 95% CI (1.73, 3.62), *P* < 0.00001, *I*^2^ = 0%, *Z* = 4.90).

### 3.4. Diagnostic Specificity Analysis of CA199

The difference in diagnostic specificity analysis of CA199 between the two groups, which was statistically significant (OR = 1.98, 95% CI (1.60, 2.44), *P* < 0.00001, *I*^2^ = 89%, *Z* = 6.35).

### 3.5. Diagnostic Sensitivity Analysis of CA199

The difference in diagnostic sensitivity analysis of CA199 between the two groups, which was statistically significant (OR = 1.92, 95% CI (1.46, 2.52), *P* < 0.00001, *I*^2^ = 73%, *Z* = 4.70).

### 3.6. Diagnostic Specificity Analysis of HE4

The total 95% CI was 2.08 (1.65, 2.63), with heterogeneity of Chi^2^ = 11.13, *P* < 0.00001, *I*^2^ = 73%, *Z* = 6.19. The difference in diagnostic specificity analysis of HE4 between the two groups was statistically significant (*P* < 0.00001).

### 3.7. Diagnostic Sensitivity Analysis of HE4

The difference in diagnostic sensitivity analysis of HE4 between the two groups was statistically significant (OR = 2.37, 95% CI (1.87, 3.00), *P* < 0.00001, *I*^2^ = 83%, *Z* = 7.19).

## 4. Discussion

Ovarian cancer has become one of the three common malignant tumors of the female reproductive system, with the highest mortality rate and threatens women's life and health seriously [25]. Among them, epithelial ovarian cancer is the most common [26]. The early symptoms of ovarian cancer are unclear [27]. Due to lack of early diagnosis, ovarian cancer is usually diagnosed at a later stage. Moreover, the survival rate of advanced ovarian cancer is far lower than that of early ovarian cancer [28]. At present, a variety of tumor markers can be used for the diagnosis of ovarian cancer, among which CA125, CA199, and HE4 have been recognized by the public and are most widely used as tumor markers, which help improve the diagnostic efficacy of ovarian cancer [29]. There have been many studies on the diagnostic value of serum CA125, CA199, HE4, and their combination in ovarian cancer, but the results are not consistent. The combination of different studies is able to complete data through appropriate analysis methods, which can reverse the shortcomings of independent study and guide clinical application [30].

The article "A Clinical Diagnostic Value Analysis of Serum CA125, CA199, and HE4 in Women with Early Ovarian Cancer: Systematic Review and Meta-Analysis" was retracted in 2023. Reasons: unreliable results or conclusions; concerns about the data; concerns about the peer review; concerns about the citations.

Therefore, we conducted literature quality evaluation and meta-analysis of independent studies [31–33] to evaluate the value of serum CA125, CA199, HE4, and their combined application in the diagnosis of ovarian cancer and to provide reliable data for clinical treatment. In the meta-score analysis, its area represents the weight assigned to the study. A larger point means a larger weight and determines a better calculation result. A horizontal line extending from the center to the two ends represents the confidence interval (CI, usually 95% CI), indicating whether there is a statistical difference between the results of individual studies [34–36]. If the 95% CI of RR OR OR of a study contains 1, as shown in the forest map, where the horizontal line of 95%C intersects the invalid line, the study can be considered to have no statistical significance. If the horizontal line falls on both sides of the vertical line without the effect, the study is considered to be statistically significant. When the horizontal line fell to the left of the invalid line, the incidence of the study was greater than that in the control group [37]. Conversely, when the incidence in a study was lower than that in the control group, the line fell to the right of the ineffective line. The combined effect sizes included in all studies are represented by the bottommost edge symbol [38, 39].

There are limitations and deficiencies of this study: (1) the search database is not extensive enough, which may lead to the omission of some literature; (2) restricting the included literature to Chinese and English might make the included research influenced by region and language, so that some studies cannot be retrieved electronically and some unpublished studies are not included, which actually increase the possibility of language bias or publication bias; (3) without manual search, some gray pieces of literature could not be obtained, such as works of literature with notable and missing data in published literature, which may cause certain publication bias in meta-analysis, and all the above reasons may lead to sampling bias in this study.

The article "A Clinical Diagnostic Value Analysis of Serum CA125, CA199, and HE4 in Women with Early Ovarian Cancer: Systematic Review and Meta-Analysis" was retracted in 2023. Reasons: unreliable results or conclusions; concerns about the data; concerns about the peer review; concerns about the citations.

## 5. Conclusion

In conclusion, the combined detection of CA125, CA199, and HE4 in this study has high diagnostic efficacy, which can improve the sensitivity and accuracy of ovarian cancer diagnosis and have certain clinical value for the diagnosis and differential diagnosis of ovarian cancer, which will provide reference significance for follow-up research and clinical decision-making.

## Figures and Tables

**Figure 1:** Flow chart of the literature screening.

**Figure 2:** Literature quality evaluation chart. (a) Risk of bias graph. (b) Risk of bias summary.

**Figure 3:** (a)–(d) Funnel plot of literature publication bias.

**Figure 4:** Meta-analysis of diagnostic specificity analysis of CA125 between two groups.

**Figure 5:** Meta-analysis of diagnostic sensitivity analysis of CA125 between two groups.

**Figure 6:** Meta-analysis of diagnostic specificity analysis of CA199 between two groups.

**Figure 7:** Meta-analysis of diagnostic sensitivity analysis of CA199 between two groups.

**Figure 8:** Meta-analysis of diagnostic specificity analysis of HE4 between two groups.

**Figure 9:** Meta-analysis of diagnostic sensitivity analysis of HE4 between two groups.

**Table 1:** Basic clinical features of 15 literature were included in our study.

Study	Age	Gender	Follow-up time (month)	The experimental group (*N*)	Control group (*N*)	NOS score	HAMD score
Liu 2017	53.71 ± 2.2	Female	3 ~ 12	52/66	15/31	8	26.12 ± 4.75
Chen 2018	55.65 ± 3.4	Female	12~24	178/262	112/386	7	23.22 ± 2.75
Simmons 2016	63.12 ± 4.5	Female	6 ~ 12	118/142	98/217	8	25.15 ± 4.02
Xiang 2017	57.15 ± 4.5	Female	6 ~24	78/133	21/43	7	23.45 ± 4.15
Rosen 2005	42.85 ± 8.4	Female	6 ~24	156/296	140/296	8	21.12 ± 4.05
Zhu 2021	64.36 ± 1.2	Female	4 ~ 12	93/179	86/179	7	28.12 ± 3.75
Cho 2019	62.62 ± 2.2	Female	6 ~ 12	50/81	31/81	9	28.21 ± 1.75
Yu 2020	62.61 ± 3.0	Female	6 ~ 18	67/102	35/102	9	27.12 ± 3.22
Xu 2021	57.25 ± 4.5	Female	6 ~24	45/75	30/75	7	29.46 ± 2.55
Freydanck 2012	56.22 ± 5.2	Female	4 ~24	32/56	24/56	8	26.42 ± 5.05
Chen 2015	61.35 ± 8.1	Female	3 ~ 12	178/323	145/323	7	24.13 ± 4.11
Chen 2017	47.25 ± 6.0	Female	4 ~ 14	98/178	80/178	7	26.16 ± 2.75
Gao 2021	58.51 ± 2.6	Female	6 ~24	40/65	25/65	9	26.18 ± 3.72
Huang 2015	66.34 ± 22.5	Female	6 ~24	48/78	30/78	8	28.16 ± 4.86
Tang 2021	62.51 ± 4.6	Female	4 ~ 12	112/190	78/190	9	25.16 ± 1.86

## Data Availability

The data used to support this study are available from the corresponding author upon request.
